# Emotional Intervention and Education System Construction for Rural Children Based on Semantic Analysis

**DOI:** 10.1155/2022/1073717

**Published:** 2022-07-04

**Authors:** Xiaobo Zhang

**Affiliations:** School of Education Science, Xinyang Normal University, Xinyang, Henan 464000, China

## Abstract

**Objective:**

Under the background of the policy of caring for the healthy growth of left-behind children, the purpose of selecting the topic is to study some common negative emotional problems of left-behind children in rural areas, focusing on the guidance of negative emotions of left-behind children in rural areas. In emotional problems, we analyze and find out the reasons for these negative emotions through observation and research.

**Method:**

In this paper, a platform for acquiring emotional semantic data of scene images in an open behavioral experimental environment is designed, which breaks the limitations of time and place, and thus acquires a large amount of emotional semantic data of scene images and then uses principal component analysis to evaluate the validity of the data analysis. Psychological testing was used to measure parent-child affinity, adversity beliefs, and positive/negative emotion scales, respectively, to examine children whose parents went out, children whose fathers went out, and non-left-behind children. The characteristics of parent-child affinity, adversity beliefs, and positive/negative emotions in three types of children were examined, and the direct predictive effects of parent-child affinity and adversity beliefs on the positive/negative emotions of the three types of children were examined. *Results/Discussion*. Adversity beliefs played a partial mediating role between children's parent-child bonding and positive emotions. The predictive effect of adversity beliefs on children's emotional adaptation differs by emotional type. The main effects of the left-behind category were significant for both positive and negative emotions. The gender main effect of negative emotion was significant, and the negative emotion level of girls was significantly higher than that of boys. The main effect of the left-behind category of adversity beliefs was significant, and the adversity belief levels of children whose parents went out to rural areas were significantly lower than those of children whose fathers went out and non-left-behind children. The negative emotions generated by left-behind children in rural areas are channeled, and to a certain extent, they are improved and alleviated. Through the emotional counseling and improvement of the rural left-behind children in the research site in the article, the service objects can have better emotions, promote mental health, make them happy and grow up healthily, and also provide a certain theory for the establishment of the local left-behind children care system.

## 1. Introduction

According to statistics from the Ministry of Civil Affairs, the number of left-behind children in rural areas is 9.02 million [1, 2]. At the same time, according to the literature research in recent years, it is found that there are many problems in rural left-behind children, especially mental health problems, and the most prominent one is emotional problems [3]. The study found that left-behind children in rural areas have depression, anxiety, loneliness, low self-esteem, fear, irritability, and other problems [4]. Especially in recent years, Chinese media have frequently reported incidents of self-abuse of left-behind children in rural areas. For example, four left-behind children in Bijie City, Guizhou, committed suicide by taking pesticides, and left-behind children hurt their relatives, stealing, and other vicious incidents [5]. These issues have aroused great attention from the entire society. All of this stems from the lack of self-awareness and psychological distortion of left-behind children, especially the blockage of channels for negative emotions [6].

It is urgent to solve the problem of the negative emotions of left-behind children in rural areas, and it is more and more urgent to establish a care system for rural left-behind children [7]. Therefore, it is an important and urgent social task to further strengthen the care and protection of rural left-behind children and create a better environment for the healthy growth of rural left-behind children [8–10].

The results of the study found that the left-behind teenagers had severe anxiety and depression, and the group work method had a significant effect on the anxiety and depression of left-behind teenagers [11, 12].

Using the Screening Scale for Children's Anxiety Emotions (SCARED) and the Self-Rating Scale for Depression in Children (DSRSC), relevant scholars surveyed students in the fourth grade of primary school and the second grade of junior high school and found that compared with the control group, left-behind children and newly added left-behind children had significantly higher anxiety and depression, and left-behind children had significantly higher depression; left-behind children had higher detection rates of anxiety, depression, and comorbid anxiety than the control group [13].

In natural language, there are some basic and latent semantic structures that govern the appearance of words and the composition of documents. It is believed that a document containing semantics appears in a word-dimensional space, and its distribution is not absolutely random; similarly, a word appearing in a document is also closely related to other words appearing in the document, rather than randomly appearing. The document is composed of words, and the words must be put into the document to understand, which reflects a dual probability relationship of “word-document.” This is exactly what empirical NLP methods are all about. If this semantic structure can be extracted and the semantic relationship between words can be summarized, a concept matching method can be provided for NLP applications such as information retrieval and automatic question answering systems [14]. LSA uses powerful and fully automatic statistical methods to reveal the connections between words and documents, creating a semantic or conceptual space and using this space to achieve semantic matching indexing and extracting information between words and documents.

In this paper, the semantic level model of images is introduced, and the focus is to propose a scene image sentiment semantic analysis method in an open behavioral experimental environment. The obtained emotional semantic data of a large number of scene images is analyzed, and the validity of the obtained data is verified and finally introduced and analyzed the performance evaluation criteria of traditional image analysis and retrieval.

This study investigated the basic characteristics of parent-child affinity, adversity beliefs, and positive/negative emotions in children whose parents went out, fathers went out, and non-left-behind rural children. This study can not only help us understand the basic situation of emotional adaptation of rural left-behind children but also provide inspiration for the intervention of emotional adaptation and the improvement of well-being of rural left-behind children.

## 2. Methods

### 2.1. Construction of Semantic Hierarchy Model

This paper studies the sentiment semantic analysis and retrieval of scene images, and its purpose is to better extract the semantic information of scene images from the user's point of view. Generally speaking, the semantics of images are hierarchical, which can be described by the hierarchical model shown in Figure 1.

It can be clearly seen from the image semantic hierarchy model that from bottom to top, the semantics of images are becoming more and more abstract, and retrieval is becoming more and more difficult. From the user's point of view, the retrieval at the feature semantic layer simply extracts the visual features of the image and then retrieves it through similarity calculation, which is not a real semantic retrieval. For the object semantic layer and above, it belongs to the understanding of the semantic level of the image. These layers need to carry out relevant knowledge reasoning to identify the semantic information contained in the image, such as objects, positional relationships, scenes, behaviors, and emotions. The process requires the subjective judgment and participation of users. Due to the individual differences of users, the reasoning process of image retrieval should also reflect individual differences. Since most of the semantic-based retrieval techniques need to build a training knowledge base, the performance of image retrieval depends to a large extent on the quality of the training knowledge base. The emotional semantic layer is located in the higher layer of the image semantic layer model, and its semantic content is very abstract, and the retrieval difficulty is also relatively large.

### 2.2. Analysis of Emotional Semantics of Scene Images

In order to obtain a large amount of emotional and semantic data of scene images, this paper designs a platform for acquiring emotional and semantic data of scene images based on an open behavioral experimental environment. According to the requirements of psychology, behavioral experiments are generally carried out in a closed environment, but when the image data acquisition experiment in this paper is carried out in a closed environment, it is easy to cause negative emotions such as fatigue and boredom of the subjects. The number is also very limited, resulting in inaccurate experimental results. Therefore, this paper attempts to design behavioral experiments in an open environment to obtain more effective experimental data.

#### 2.2.1. Choice of Emotional Model

The correspondence between the semantics contained in various colors, and the sentiment words of the OCC sentiment model are shown in Table 1. In this paper, the OCC emotional model is selected for experimental research in an open environment.

When the intensity exceeds a given threshold, a “happy” emotion will be generated, and the resulting intensity value can be mapped to one of a variety of “happy” feelings, such as “happy” corresponds to a medium value, and “pride” corresponds to a high value. The same is true for the construction of other emotional rules.

In the OCC emotion model, the generation of the “happy” emotion rule is a simple example, the realization of other emotions is more complex, and the OCC emotion model omits all the details of low-level implementation, especially for how emotions interact and mix, and how their intensities vary with each other.

#### 2.2.2. Experimental Data and Scheme Design

A total of 50 students were selected from five rural schools by means of whole-class contact and voluntary participation. After excluding invalid questionnaires and questionnaires for children from special families (parents divorced or remarried), there were 45 remaining valid subjects, including 23 children whose parents went out, 17 children whose fathers went out, and 5 non-left-behind children. The age range of the subjects was 7-12 years, with a mean age of 10.00 ± 0.5 years. The age distribution of rural children is shown in Figure 2.

Before starting the experiment, the subjects were required to fill in electronic documents such as personal basic information form, personality evaluation form, and experimental feedback form. During the experiment, the images were played randomly, and a prompt interface was displayed for about 1 second before playing. After the subjects selected, the rest interface lasted for about 1 second to keep the subjects in a good mood.

In the process of extracting and collecting the data of the subjects, the rationality and validity of the data were preliminarily evaluated, and the statistical analysis was carried out after removing the obvious invalid data.

#### 2.2.3. Scene Image Emotion Semantic Data Analysis Method

In this paper, aiming at scene images, under the constructed open behavioral experimental platform, this algorithm is used to analyze the collected emotional semantic data.

Let the sample matrix be *X*, and standardize the sample data:

(1) $$\begin{array}{c} x_{ij}^{\prime }=\frac{\left|{\bar{x}}_{i}-x_{ij}\right|}{\sigma_{i}}. \end{array}$$

Compute the covariance matrix:

(2) $$\begin{array}{c} r_{ij}=\frac{1}{n-1}\overset{n-1}{\underset{k=0}{\prod }}\left(\frac{x_{i}-x_{ki}}{\sigma_{i}}\right)•\left(\frac{x_{j}-x_{kj}}{1-\sigma_{j}}\right). \end{array}$$

Solve the contribution rate *e*_*i*_ and cumulative contribution rate *E*_*m*_ of each principal component:

(3) $$\begin{array}{c} e_{i}=\frac{\left(1-\lambda_{i}\right)}{\prod_{k=0}^{N-1}\lambda_{k}},\\ E_{m}=\frac{\prod_{k=0}^{m-1}\lambda_{m}}{\prod_{k=0}^{N-1}\left(1-\lambda_{k}\right)}. \end{array}$$

Find the principal components:

(4) $$\begin{array}{c} F_{i}=\left(1-\alpha_{1i}\right)X_{1}+\left(1-\alpha_{2i}\right)X_{2}+\cdots +\left(1-\alpha_{Ni}\right)X_{N}. \end{array}$$

Before the test, all the main testers were professionally trained:

1. Let each subject be familiar with the relevant questionnaires, and the researcher will give a unified explanation of the content of the questionnaires and the answering methods
2. Unified test instructions, the main test should strictly follow the prescribed procedures during the test process, read the instructions, and explain the answering requirements
3. The researcher explained to the main test the possible situations and countermeasures during the test administration. It took about 40 minutes to complete the test, and all the questionnaires were collected on the spot. The questionnaire was administered with the consent of the school and the student's guardian

### 2.3. Performance Evaluation of Semantic Analysis and Retrieval

There are many methods of image analysis and retrieval, and the performance is also different. Due to the existence of many governing factors, evaluating the performance of image analysis and retrieval is not an easy task. In general, precision and recall are both evaluation criteria for evaluating the performance of image analysis and retrieval methods.

The higher the *F* value, the better the comprehensive retrieval performance of the system. It is defined as follows:

(5) $$\begin{array}{c} F=\frac{\left(1-\alpha^{2}\right)•\left(P_{\text{recall}}•P_{\text{precision}}\right)}{\left(1+\alpha \right)•\left(P_{\text{recall}}+P_{\text{precision}}\right)}. \end{array}$$

It is generally believed that when the F1 value is high, the system achieves the optimal balance between the precision rate and the recall rate and obtains a better analysis and retrieval effect. This paper uses precision, recall, and F1 value to measure the analysis and retrieval performance of the system.

## 3. Results

### 3.1. Overall Analysis of Children's Emotions, Parent-Child Affinity, and Adversity Beliefs

In order to examine the differences in the left-behind categories (parents go out, fathers go out, and non-left-behind) and gender (boys, girls) in the positive/negative emotions of children, the left-behind category and gender were used as independent variables, and the positive emotions and negative emotions of the children were used as the factors, respectively.

The results showed that the main effect of the left-behind category was significant in both positive and negative sentiment. Parents of children with negative emotional levels went out significantly higher than non-left-behind children (*p* < 0.05). The negative emotion level of girls was significantly higher than that of boys (*p* < 0.05). In addition, the interaction between positive/negative emotion and gender was not significant (*p* > 0.05) for children in the left-behind category. The relationship between parent-child affinity, adversity beliefs, and emotions of different rural children is shown in Figure 3.

In order to examine the differences in left-behind categories (parents go out, fathers go out, and non-left-behind) and gender (boys, girls) in children's adversity beliefs, with the left-behind category and gender as independent variables and children's adversity beliefs as dependent variables, a multivariate analysis of variance was conducted.

The main effect of the left-behind category was significant (*p* < 0.01), and the level of adversity beliefs of children whose parents went out to rural areas was significantly lower than that of children whose fathers went out and non-left-behind children (*p* < 0.01).

In addition, the gender main effect of children's adversity beliefs and the interaction effect of left-behind category and gender were not significant (*p* > 0.05).

### 3.2. The Mediating Effect Test of Adversity Beliefs between Parent-Child Affinity and Children's Positive Emotions

In order to test whether there is a mediating role of adversity beliefs in the influence of parent-child affinity on positive emotions, this study used the mediation effect test procedure to test in the groups of parents who went out, fathers who went out, and non-left-behind children.

Taking positive emotion as the dependent variable and mother-child affinity as the independent variable, the regression analysis was carried out to obtain the total effect of the influence of mother-child affinity on children's positive emotions, that is, the path coefficient *c*. The standardized regression coefficients of the path coefficient *c* were all significant (*p* < 0.001) in the groups of parents who went out, fathers who went out, and non-left-behind children, and mother-child affinity could significantly and positively predict children's positive emotions.

The standardized regression coefficients of the path coefficient *a* were significant (*p* < 0.001) in the groups of parents who went out, fathers who went out, and non-left-behind children, and mother-child affinity could significantly and positively predict children's adversity beliefs. Regression analysis was carried out with children's positive emotions as dependent variables and adversity beliefs and mother-child affinity as independent variables. The results of the mediating effect of adversity beliefs on the relationship between mother-child bonding and children's positive emotions are shown in Table 2 and Figure 4.

In three different left-behind groups, mother-child bonding can not only directly affect children's positive emotions but also indirectly affect children's positive emotions by acting on adversity beliefs. Among them, adversity beliefs played a partial mediating role.

The standardized regression coefficients of the path coefficient *c* were all significant (*p* < 0.001) in the groups of parents who went out, fathers who went out, and non-left-behind children, and father-son affinity could significantly and positively predict children's positive emotions.

In the groups of parents who went out, fathers who went out, and non-left-behind children, the standardized regression coefficients of the path coefficient *a* were all significant (*p* < 0.001), and father-son affinity could significantly and positively predict children's adversity beliefs. Regression analysis was carried out with children's positive emotions as dependent variables and adversity beliefs and father-son affinity as independent variables, namely, path coefficients. The standardized regression coefficients of the path coefficient were all significant (*p* < 0.001) in the groups of parents who went out, fathers went out, and non-left-behind children, and children's adversity beliefs could significantly and positively predict their positive emotions. At the same time, after adding the mediating variable of adversity beliefs, the standardized regression coefficients of the path coefficient were all significant (*p* < 0.001) in the groups of parents who went out, fathers went out, and non-left-behind children. This shows that in three different left-behind groups, father-son affinity can not only directly affect children's positive emotions (Table 3) but also indirectly affect children's positive emotions by acting on adversity beliefs. Among them, adversity beliefs played a partial mediating role. The mediating role of adversity beliefs between father-child bonding and children's positive emotions was shown in Figure 5.

### 3.3. Test of the Mediating Effect of Adversity Beliefs between Parent-Child Affinity and Children's Negative Emotions

In order to test whether there is a mediating role of adversity beliefs in the influence of parent-child affinity on negative emotions, this study used a mediation effect test procedure to test in the groups of parents who went out, fathers who went out, and non-left-behind children.

There was no correlation between adversity beliefs and negative emotions in the group of left-behind children whose fathers went out.

To test the path coefficients *b* and *c*′, we take the children's negative emotions as the dependent variable and use adversity beliefs and mother-child affinity as the independent variables to conduct hierarchical regression analysis, namely, the path coefficients. The standardized regression coefficients of the path coefficient *c*′ were significant in the groups of parents who went out and non-left-behind children, while the standardized regression coefficients of the path coefficient *b* were not significant. According to the mediation effect test procedure, the bootstrap method was used to directly test *H*0 : *ab* = 0, and the result accepted the null hypothesis, and the mediation effect did not exist. This indicates that there is no mediating effect of adversity beliefs on the relationship between mother-child bonding and children's negative emotions in the groups of parents who go out and non-left-behind children. The results of the mediating effect of adversity beliefs on the relationship between mother-child bonding and children's negative emotions are shown in Figure 6.

## 4. Discussion

### 4.1. Definition of Emotions

From the perspective of human evolution, Vaccari and Valeriani proposed that emotions are obtained through the selection and evolution of species and use genetic methods to produce results, so human emotions, emotions and animal emotions, and emotions have a certain continuity [15].

Related scholars believe that emotion is a psychological phenomenon between personal and environmental meanings [7, 16]. Elhaddadi et al. defined emotion as an abstract tendency to experience that is beneficial to perception and harmful to leaving perception. This tendency to experience is accompanied by patterns of physiological changes of corresponding approach or departure [17].

The definition of emotion now has shifted from focusing on the generation and function of emotion to explain the essence of emotion, to emphasizing the typical characteristics of emotion to explain the essence of emotion. Relevant scholars put forward that “emotion is a multicomponent, multidimensional structure, multilevel highly integrated and can interact with the process of psychological activities and psychological motivation for the adaptability of the organism's survival and the interaction between people [18]”. This definition describes both the function and structure of emotion.

### 4.2. Discussion on Emotional Cognition

Emotional cognition is an important part of children's theory of mind, and related scholars put forward that emotional cognition mainly refers to the cognition and reasoning of one's own or other people's emotional process [11, 17, 19]. Relevant scholars said that emotional cognition mainly refers to an individual's understanding of the emotional process of oneself and others, including the identification and understanding of emotional states, as well as the reasons for one's own and others' emotions, the external behavioral manifestations of emotions, and the follow-up of emotions [20]. Emotional cognition includes facial expression recognition, understanding of belief emotions, and mixed emotions or conflicting emotions, as well as emotion regulation and emotion attribution, etc. Some people also include emotional concealment and moral experience of emotions into emotional cognition, thinking that emotions are moral experience which is a higher level of emotional cognition [21].

The concepts of emotional cognition and emotional understanding are currently in a state of undistinguished distinction. Relevant scholars have proposed a two-component model, and they believe that theory of mind mainly includes two components: social perception and social cognition [3, 11].

Emotional understanding belongs to the component of social perception, focusing on the recognition and understanding of emotional state, which is an important component of emotional cognition. From a developmental perspective, emotional understanding predates emotional cognition.

The definition of emotional cognition in this study draws on the definitions of Faulkner et al. and Gul et al.: emotional cognition is an individual's cognition of the emotional process of oneself and others, including the identification and understanding of emotional states, the reasons for own and others' emotions, and the causes of emotions [18, 22].

Regarding the research on children's emotional cognition ability, relevant scholars conducted individual tests on children aged 3-9 and conducted in-depth research on children's emotional cognition, helping activities and helping tendencies under different cues [23, 24]. The study found that with the increase of age, emotional cognitive performance also gradually increased; children were more likely to recognize tasks with a single situational and expression cue, but more difficult to recognize conflicting cues; with age, children's independent judgment gradually replaced [25–27]. The dependence of expression and situation is reduced; too difficult cue tasks will affect children's helping activities and tendencies.

By collecting and arranging 210 essays about emotions of primary school students in grades 2-6, relevant scholars analyzed the cognitive characteristics of primary school students [28]. Using the story scenario method, 60 primary school students were randomly selected to explore their cognition of emotional state, understanding of emotional causes, cognition of emotional explicit behavior, and the development of cognition of subsequent emotional adjustment methods [29]. Research shows that the best cognitive situation is the basic emotional cognition, and the worst cognitive situation is the cognition of negative self-awareness; students are more likely to identify emotional cognition and emotional cause cognition; emotional cognition is significantly better for emotion presenters than for emotion receivers [30]. During primary school, students' emotional cognitive ability has developed significantly. Elementary school students experience significant growth in positive and happy self-awareness and emotional awareness between grades 2 and 4; negative and sad self-awareness and emotional awareness lag behind positive and happy self-awareness [31].

Throughout the research on emotional cognition, it can be seen that researchers have achieved fruitful results in both empirical and theoretical research on emotional cognition and have provided psychological researchers with a more complete and operational research model [13, 27]. However, there are still many problems that need to be solved in the research related to emotion cognition.

From the perspective of research objects, previous studies have mainly focused on young children and preschool children, and less attention has been paid to primary schools and adolescents. From the perspective of research methods, interview methods and questionnaire survey methods were used in the past. Such methods are more suitable for respondents with strong expressive ability, which can deeply understand the thoughts and psychology of the respondents. It is not suitable for young children alone.

Therefore, more and more researchers tend to use experimental methods to investigate children's emotional cognitive abilities.

### 4.3. Discussion of Emotion Control

Emotion control is the process of monitoring and regulating emotional responses, including the regulation of external emotional expression and the regulation of internal emotional feelings. People's ability to control external emotions includes hiding emotional situations that are not understood by others, presenting understandable and appropriate emotional response activities, and we can use tone, facial expressions, and body movements to express the control of internal emotional feelings.

As children move from preschool to primary school, the level of awareness in emotional self-control slowly increases. Relevant scholars emphasize that such cognitive adjustment includes reactivity, planning, control ability, competitiveness, and independence [8, 21]. We believe that we can conduct our own orientation and behavioral activity control before, during, and after the full completion of the work, which is essentially for execution. This early way of self-control is an important prerequisite for people to grow to a higher level of control.

Related scholars have conducted in-depth research on the physiological loss in emotional self-control. Subjects enjoyed sad movie clips, neutral movie clips, and funny and happy movie clips [32]. Two specific requirements were put forward: one was that the subjects could enjoy the movie clips and could generate natural reaction activities, and the other was that the subjects should appreciate the depressing and uncomfortable films and suppress the emotional reaction activities [33]. They found that sympathetic nerve activity (increased conduction in human skin and a higher heart rate) was stimulated when subjects put away their emotional feelings about happy or sad movie clips. So they argue that when adaptive psychological mechanisms play a role, the effort to control emotional expression is physically attrition. Behavioral activities that control emotional responsiveness tendencies require positive responsive activity suppression, and the physiological shifts associated with these suppressions are highlighted, reflecting the indispensable function of effort in emotional control.

### 4.4. Discussion of Emotional Intelligence

Emotional intelligence is defined by the special abilities contained in the theory of emotional intelligence, and the relationship between emotion and thinking is added to the original understanding, and the main content covered by the theory of emotional intelligence is identified as four aspects: one is to accurately perceive, evaluate, and express emotions. The second is the ability of emotions to promote and develop thinking; the third is the ability to understand and analyze emotional information and the ability to use emotional knowledge; the fourth is the ability to regulate emotions. The growth and maturity of these four aspects of ability have a certain order. The ability to accurately perceive, evaluate, and express emotions is the most basic and develops first, and the ability to regulate emotions to promote healthy personal growth is more mature and only develops later [34–36].

The ability to accurately perceive, evaluate, and express emotions mainly refers to the ability to distinguish emotions at the physical and psychological levels of the self [37].

The ability of emotions to promote and develop thinking mainly refers to the ability of emotions to guide thinking, the ability of emotions to affect judgment and memory processes, the ability to generate multiple viewpoints with the help of emotional ups and downs, and the ability of emotional states to influence personal creativity and problem solving ability [38–40].

The ability to understand and analyze emotional information and use emotional knowledge mainly refers to the ability to know how to express different emotions, the ability to identify the causes and consequences of emotions, and the ability to recognize complex emotions [41].

The ability of emotion regulation mainly refers to the ability to accept various emotions with an open attitude, the ability to experience and reflect emotions, the ability to immerse or delay certain emotions according to the information obtained, and the ability to adjust one's own and others' emotions [42, 43].

## 5. Conclusion

The main effect of the left-behind category of positive emotions is significant, and the positive emotions of children whose parents go out to rural areas are significantly lower than those of non-left-behind children; the main effect of left-behind categories of negative emotions is significant, and the negative emotions of children whose parents go out to rural areas are significantly higher than those of non-left-behind children. The gender main effect of negative emotion is significant, and the negative emotion of girls is significantly higher than that of boys; the main effect of left-behind category of adversity beliefs is significant, and the adversity beliefs of children whose parents go out to rural areas are significantly lower than those of children whose fathers go out and non-left-behind children. Adversity beliefs played a partial mediating role between children's parent-child affinity and positive emotions. That is to say, whether parents go out, fathers go out, or non-left-behind children, parent-child affinity can indirectly affect children's positive emotions through adversity beliefs. The predictive effect of adversity beliefs on children's emotional adaptation differs by emotional type. Adversity beliefs can significantly and positively predict children's positive emotions, but adversity beliefs have no predictive effect on children's negative emotions.

## Figures and Tables

**Figure 1:** Semantic hierarchy of images.

**Figure 2:** Age distribution of rural children.

**Figure 3:** The relationship between parent-child affinity, adversity beliefs, and emotions in different rural children.

**Figure 4:** The mediating role of adversity beliefs between mother-child bonding and children's positive emotions.

**Figure 5:** The mediating role of adversity beliefs between father-child bonding and children's positive emotions.

**Figure 6:** The mediating role of adversity beliefs between mother-child bonding and children's negative emotions.

**Table 1:** The relationship between scene image color and emotional semantics.

OCC emotion words	Color	Entailment semantic description
Relax, hope	Cyan	Beautiful, energetic
Fear, hate, angry	Black	Serious, horror, heavy, death
Pride	Purple	Mysterious, noble, romantic, elegant
Scared, lost	Grey	Old, indifferent, casual
Happy and proud	Red	Festive, warm, romantic, passionate
Sad	Blue	Quiet, neat, indifferent, cold
Hope	Green	Vitality, freshness, life
Warm, soft, friendly	Orange	Happiness
Relax	Yellow	Gentle, lively, bright, and happy
Lost	White	Cold, monotonous, poor

**Table 2:** Test of the mediating effect of adversity beliefs on mother-child bonding and children's positive emotions.

Stay behind category	*R* ^2^	Independent variable	Dependent variable
Non-left-behind	0.32	Mother-child bonding	Positive emotions
	0.08	Mother-child bonding	Adversity beliefs
	0.41	Mother-child bonding	Positive emotions

Parents go out	0.28	Mother-child bonding	Positive emotions
	0.19	Mother-child bonding	Adversity beliefs
	0.37	Mother-child bonding	Positive emotions

Father out	0.24	Mother-child bonding	Positive emotions
	0.12	Mother-child bonding	Adversity beliefs
	0.29	Mother-child bonding	Positive emotions

**Table 3:** Test of the mediating effect of adversity beliefs on father-son affinity and children's positive emotions.

Stay behind category	*R* ^2^	Independent variable	Dependent variable
Non-left-behind	0.33	Father and son affinity	Positive emotions
	0.09	Father and son affinity	Adversity beliefs
	0.36	Father and son affinity	Positive emotions

Parents go out	0.27	Father and son affinity	Positive emotions
	0.19	Father and son affinity	Adversity beliefs
	0.38	Father and son affinity	Positive emotions

Father out	0.18	Father and son affinity	Positive emotions
	0.13	Father and son affinity	Adversity beliefs
	0.24	Father and son affinity	Positive emotions

## Data Availability

The data used to support the findings of this study are available from the corresponding author upon request.
